# Identification of the Mechanism of Matrine Combined with Glycyrrhizin for Hepatocellular Carcinoma Treatment through Network Pharmacology and Bioinformatics Analysis

**DOI:** 10.1155/2022/2663758

**Published:** 2022-09-19

**Authors:** Tao Han, Yiming Liu, Yutong Chen, Tingsong Chen, Yifan Li, Qiuhua Li, Mingfang Zhao

**Affiliations:** ^1^Department of Medical Oncology, The First Hospital of China Medical University, Shenyang, Liaoning 110000, China; ^2^Liaoning University of Traditional Chinese Medicine, Shenyang, Liaoning 110000, China; ^3^The General Hospital of Northern Theater Command Training Base for Graduate, China Medical University, Shenyang, Liaoning 110000, China; ^4^Department of Oncology, Shanghai Seventh People's Hospital, Shanghai 200137, China; ^5^The First Department of Clinical Medicine, China Medical University, Shenyang, Liaoning 110000, China

## Abstract

Matrine and glycyrrhizin are representative active ingredients of traditional Chinese medicine (TCM) used in clinical practice. Studies have demonstrated that matrine has antitumor pharmacological effects and that glycyrrhizin protects liver function. However, the potential bioactive compounds and mechanisms remain unknown, as well as whether they have synergistic effects in killing cancer cells and protecting liver cells. To investigate the synergistic effects and mechanism of matrine combined with glycyrrhizin in hepatocellular carcinoma (HCC) treatment, we used both network pharmacology and bioinformatics analyses. First, the chemical gene interaction information of matrine and glycyrrhizin was obtained from the PubChem database. The pathogenic genes of HCC were accessed from five public databases. The RNA sequencing data and clinical information of HCC patients were downloaded from The Cancer Genome Atlas (TCGA). Next, the overlapping genes among the potential targets of matrine and glycyrrhizin and HCC-related targets were determined using bioinformatics analysis. We constructed the drug-target interaction network. Prognosis-associated genes were acquired through the univariate Cox regression model and Lasso-Cox regression model. The results were verified by the International Cancer Genome Consortium (ICGC) database. Finally, we predicted the immune function of the samples. The drug-target interaction network consisted of 10 matrine and glycyrrhizin targets. We selected a Lasso-Cox regression model consisting of 3 differentially expressed genes (DEGs) to predict the efficacy of the combination in HCC. Subsequently, we successfully predicted the overall survival of HCC patients using the constructed prognostic model and investigated the correlation of the immune response. Matrine and glycyrrhizin have synergistic effects on HCC. The model we obtained consisted of three drug-target genes by Lasso-Cox regression analysis. The model independently predicted the combined effect of matrine and glycyrrhizin in HCC treatment and OS, which will be helpful for guiding clinical treatment. The prognostic model was correlated with the immune cells and immune checkpoints of patients, which had an adjuvant effect on HCC immunotherapy. Matrine and glycyrrhizin can have therapeutic effects on HCC by promoting the production or enhancing the core gene activity in the drug network and improving the immune system function of patients.

## 1. Introduction

HCC is a malignant tumor that seriously threatens human life and health. According to 2020 oncology epidemiology data, the mortality rate of HCC is very high, and HCC has become the second leading cause of cancer-related death after lung cancer [1], and most patients are diagnosed and treated at the clinical III or IV stage [2]. Thus, the treatment of HCC has become a medical challenge worldwide. Treatment approaches include radiation, transplant, and surgery. In recent years, systematic therapies such as targeted and immune therapy have made important progress in the treatment of advanced liver cancer. Targeted therapy for HCC mainly includes multikinase inhibitors (TKIs) and antiangiogenic drugs, such as sorafenib, lenvatinib, donafenib, regorafenib, and apatinib, while immune checkpoint inhibitors are used in immunotherapy treatment [3]. With the wide application of ICIs in the treatment of hepatocellular carcinoma, the toxic side effects caused by ICI activation, namely, immune-related adverse reactions (irAEs), have become a major challenge in clinical practice [4]. Currently, the objective of therapy for liver cancer is to prolong overall survival. However, the benefits of TCM treatments seem to be promising in liver cancer [2], breast cancer [5], etc. Thus, clarifying the anticancer mechanism of action of TCM treatment is important. Wu et al. investigated the mechanism of a Bushen-Jianpi decoction (BSJPD) in liver cancer (LC) treatment [6]. Correlation analysis revealed that BSJPD was an independent protective factor for survival. They further investigated the mechanism of action of BSJPD with network pharmacology analysis and experimental verification. In this work, they identified 143 compounds in the 9 herbs of BSJPD and 249 related targets. In view of the results of the enrichment analysis, we found that the liver cancer signaling pathways impacted by treatment with BSJPD mostly involved tumor apoptosis and growth, such as the PI3K-Akt-mTOR, p53, TNF, and VEGF pathways [7, 8]. Overall, this work proves that BSJPD can prolong the survival of patients with liver cancer and promote hepatoma cell apoptosis, which is associated with its modulation of the PI3K-Akt-mTOR pathway and the p53, CASP3, and Bcl-xL/BAD proteins. These effects may be partly derived from licochalcone A, alisol B, and hederagenin, which are the 3 major compounds in the network pharmacology prediction.

Network pharmacology is the next paradigm in drug discovery [9]. The dominant paradigm in drug discovery is the concept of designing maximally selective ligands to act on individual drug targets. However, many effective drugs act via modulation of multiple proteins rather than single targets. Advances in systems biology are revealing a phenotypic robustness and network structure that strongly suggests that exquisitely selective compounds, compared with multitarget drugs, may exhibit lower than desired clinical efficacy [10–12]. This new appreciation of the role of polypharmacology has significant implications for tackling the two major sources of attrition in drug development—efficacy and toxicity. Integrating network biology and polypharmacology holds the promise of expanding the current opportunity space for druggable targets [11, 13, 14].

CHM, an ancient treatment methodology popular in China and surrounding areas, has been recognized as a pharmaceutical area of TCM and holds promise for preventing diseases in a holistic way [15, 16]. It has been used in clinical practice for a long period, and it is known for its effectiveness and beneficial contribution to public health and disease control. However, the pharmacological mechanisms of CHM have not been fully established. With increasing knowledge of the network of genes and molecular interactions, researchers have adopted network pharmacology for their drug research and development.

Building a CHM database is critical for a network pharmacology study [17]. The TCMGeneDIT database mainly focuses on TCM-related gene and disease information [18]. The TCM Database@Taiwan is applied to CHM screening [19]. There are also disease-drug-target databases used for drug-target research on herbal compounds, such as SuperTarget, Matador [20], DrugBank [21], and Therapeutic Target Database [22]. Li proposed a methodology termed “network target,” which is used to reveal the interactions between herbal compounds/formulas and complex syndrome systems based on network pharmacology and systems biology [23]. Relevant technology can be used to screen effective herbal substances and discover drug targets. Such technology could also provide theoretical support for detecting new pharmacological effects of Chinese compound formulas [17]. Essentially, the network visualization of the CHM literature examines the database to find modes or rules [24], detects the literature information, analyzes the selection data, and discovers the novel effects of CHM.

The NIMS approach could be beneficial for analyzing the therapeutic effects of multicomponent CHM. To discover the relationship between Chinese herbal multicomponent and potential pharmacological function, Li et al. applied a network target-based identification of multicomponent synergy (NIMS) algorithm to calculate the components of CHM and demonstrate the synergistic correlation of the multicomponent [25]. Fan et al. used the network pharmacology method to reconstruct the network model to describe the toxicological properties, which offered valuable information to identify the toxic substances and potential toxicity of known compounds in a complex system [26].

The characteristics of TCM theory involve the consideration of organic wholeness and treatment based on TCM syndrome differentiation. A diagram is proposed to describe the research approach of network pharmacology for CHM. This approach is a combination from the “disease-syndrome-CHM” model, which comprises the core values for reflecting disease and TCM syndrome as well as correlates with CHM, TCM syndrome, and multitarget effects. By integrating the chemical predictor, target predictor, and network building, a system of TCM was constructed. It systematically revealed the potential mechanisms of TCM [27]. The appropriate cellular and animal models are conducive to evaluating the effectiveness of TCM [28], which could be used to verify the results of network analysis and mutual authentication. However, the systemic characterization is still unclear for the drug-target correlation of CHM. Network pharmacology could be helpful to confirm the effective ingredients and promote drug discovery of CHM. Network pharmacology has become a helpful tool in understanding the fine details of drug-target interactions.

To broaden the idea of drug development, this study investigated the mechanism of the combination of traditional Chinese herb *Sophora flavescens* extract (matrine) and *Glycyrrhiza uralensis* extract (glycyrrhizin) against HCC [29, 30]. To better explore the relationship between multicomponent and target sites of TCM, we adopted the concept of network pharmacology, which facilitated our study of the complex network of TCM extracts. Matrine injection is often used as a routine drug against hepatitis virus, and glycyrrhizin is commonly used as a drug to protect liver function in clinical practice [31, 32]. The two drugs are often combined in clinical practice. Previous studies have shown that the combination of matrine and glycyrrhizin enhances the drug's efficacy and reduces the side effect of glycyrrhizin, which causes sodium and water retention [33]. However, the specific cellular pathways through which the two drugs act have not been clarified. In this study, we constructed a drug-targeting network of matrine and glycyrrhizin on hepatocarcinogenic genes by network pharmacology and screened the core genes in the network. Based on our study results, we can provide a better understanding of the interaction between the two drugs and provide basic theoretical support for future research. A core drug-target network consisting of 10 target genes was ultimately obtained. We analyzed the differential expression of transcriptomic genes in HCC and normal tissue specimens, to better predict the survival of HCC patients treated with matrine and glycyrrhizin and to facilitate clinical medication strategies. Univariate Cox regression analysis was performed on 7 DEGs in the drug-target network, and 4 DEGs with prognostic significance were finally obtained. The Lasso-penalized Cox regression analysis algorithm was used to analyze the four DEGs. Finally, we obtained a Lasso-Cox prognostic regression model composed of three differentially expressed drug-target network genes, and a prognostic nomogram was established to facilitate clinical guidance. Moreover, gene set enrichment analysis (GSEA) was performed to investigate the role of model core genes in tumorigenesis, tumor progression, and immune response. In this study, to investigate the immune-related effects of matrine and glycyrrhizin, immune cells and immune checkpoints in HCC specimens were predicted. In addition, we investigated the correlation between risk values and immune cells and immune checkpoints and further explored the effect of matrine and glycyrrhizin on the immune response.

## 2. Materials and Methods

### 2.1. Data Collection

First, the chemical gene interaction information of matrine and glycyrrhizin, including 27 matrine target information and 64 glycyrrhizin target information, was downloaded from the PubChem database (https://pubchem.ncbi.nlm.nih.gov) [34]. Hepatocarcinogenic genes were obtained from the GeneCards database (https://www.genecards.org/), Online Mendelian Inheritance in Man (OMIM) database (https://omim.org/), Pharmacogenetics and Pharmacogenomics Knowledge Base (PharmGkb) (https://www.pharmgkb.org/), DrugBank database (https://www.drugbank.com/), and Therapeutic Target Database (TTD) database (http://db.idrblab.net/ttd/). The transcriptome data and clinical data of HCC samples originated from the TCGA GDC (https://portal.gdc.cancer.gov/) database [35]. A total of 424 transcriptomic data and 377 clinical data were obtained. Transcriptomic data included all gene transcription and expression level information of the samples, and clinical data included overall survival time, survival status, age, sex, clinical stage, and other clinically relevant information. We obtained 442 transcriptome data and clinical data of HCC samples provided by RIKEN and JP from the ICGC database and the ICGC database [36]. Immunohistochemical section images of gene expression in cancer and paracancerous tissues were obtained from the Human Protein Atlas database (HPA database, https://www.proteinatlas.org/).

### 2.2. Drug-Target Interactional Network Construction and Screening

The action targets of matrine and glycyrrhizin obtained from PubChem were combined as drug targets. The HCC pathogenicity genes obtained from five disease gene databases were combined as pathogenicity genes. A protein–protein interaction (PPI) network was constructed by the STRING (https://string-db.org/) database, using the overlapping genes between the drug targets and pathogenicity genes, with a confidence interval of 0.9, and isolated genes that did not interact with other genes were eliminated. Then, the PPI network was processed with Cytoscape version 3.8.2 and screened twice using the CytoNCA plug-in in Cytoscape. Finally, the network core genes were obtained. The screening criteria were betweenness centrality (BC), degree centrality (DC), closeness centrality (CC), eigenvector centrality (EC), local average connectivity (LAC), and network centrality (NC). Both filters were based on all criteria values greater than the median.

### 2.3. Drug-Target Network Gene Function and Functional Enrichment Analysis

To explore which gene functions and cellular pathways are enriched in network core genes, Kyoto Encyclopedia of Genes and Genomes (KEGG) and Gene Ontology (GO) analyses were performed using the “clusterProfiler” R package [37]. The pathways were regarded to be significantly enriched when *P* < 0.05.

### 2.4. Differentially Expressed Gene Analysis

The expression levels of the network core genes were extracted from the transcriptome data of the TCGA database. The gene expression level heatmap was plotted by tumor group and normal group, and the gene expression association map was also drawn.

### 2.5. Construction of the Lasso-Cox Regression Prediction Model

The prognostic value of the network core genes was determined by univariate Cox regression analysis, where *P* < 0.05 was considered statistically significant. Least absolute shrinkage and selection operator- (Lasso-) penalized Cox regression analysis with the “glmnet” R package [38], was used to further identify genes relevant to the prognosis of HCC. Patients were divided into low-score and high-score groups according to the median value. The Kaplan–Meier survival curves were generated to evaluate the predictive performance of related risk genes.

### 2.6. Validation of the Lasso-Cox Regression Prediction Model

We validated this model by examining the hepatocellular carcinoma transcriptome and clinical data from the ICGC database of the RIKEN Institute of Japan (RIKEN, JP). We established a receiver operating characteristic (ROC) curve using the “timeROC,” “survival,” and “survminer” R packages to verify the model prediction performance. We generated the risk curve, risk and survival scatter plot, and heatmap of model gene expression using the “pheatmap” R package. We established a nomogram using the “rms” R package to predict the survival of patients. Based on univariate and multivariate Cox regression analyses, forest plots were drawn.

### 2.7. Correlation between the Prognostic Model and Tumor Immunity

To explore the effect of the risk score on the immune response in the Lasso regression prediction model, we downloaded the immune cell content data from the TIMER2.0 online immune database and mapped box plots and correlation plots of immune cell content. To explore the correlation between the risk score and immune cells in the Lasso regression prognostic model, we mapped the correlation plots of risk scores and various immune cells. We also explored the relationship between the risk score and immunotherapy, plotting the correlation plots between the risk scores and immune checkpoints.

## 3. Results

### 3.1. Construction of Drug-Target Interaction Networks

The mechanism by which the combination of matrine and glycyrrhizin treats HCC is a complex multicomponent and multitarget process. In this study, we used the research concept of network pharmacology. We obtained the known drug targets of matrine and glycyrrhizin from the PubChem database, as well as the interactions and effects of the corresponding drugs on the target.

Considering that obtaining data from a single disease gene database may lead to gene data loss, in this study we downloaded and combined disease-associated gene data from five disease-associated gene databases (Figure 1(a)), making the data more comprehensive and general. A total of 16937 disease-causing gene data associated with liver cancer were obtained.

There were 93 overlapping genes between the targets of matrine and glycyrrhizin and HCC pathogenicity genes (Figure 1(b)). The overlapping genes represent targets for the combined application of matrine and glycyrrhizin for the treatment of hepatocellular carcinoma. Matrine and glycyrrhizin produce specific pharmacological effects on pathogenicity genes and thus are effective in the treatment of HCC. We also created a drug-target interaction network diagram (Figure 1(c)). with a confidence interval of 0.9, and isolated genes that did not interact with other genes were eliminated. We queried and screened the interaction relationships between target proteins by the STRING online database to obtain a protein interaction network (PPI, Figure 1(d)) containing 73 target proteins (CI = 0.90), hiding independent proteins that have no interaction relationships with other proteins. We generated the interaction network of matrine and glycyrrhizin on target genes by importing the interaction information into Cytoscape version 3.8.2 (Figure 1(e)).

The protein interaction network of 93 overlapped genes was screened twice using the plug-in CytoNCA with the following criteria: BC (betweenness centrality), DC (degree centrality), CC (closeness centrality), EC (eigenvector centrality), LAC (local average connectivity), and NC (network centrality). EC, LAC, NC, and both filters were based on the condition that all criteria values were greater than the median. We finally obtained a core drug-target interaction network consisting of 10 core genes (Figure 1(f)): *TP53*, *CASP8*, *MAPK1*, *MAPK3*, *MYC*, *NFKB1*, *TNF*, *IL6*, and *NFKBIA*.

### 3.2. Gene Ontology (GO) and KEGG Pathway Enrichment Analyses

To elucidate the underlying pathways that were associated with the 10 core genes of the drug-target network, GO gene function enrichment analyses and KEGG cellular pathway enrichment analyses (Figures 2(c) and 2(d)) were performed. This study suggests that matrine and glycyrrhizin are enriched in the function of genes such as “cellular response to biological stimuli,” “cellular response to tumor necrosis factor,” “response to tumor necrosis factor,” “response to lipopolysaccharide,” “response to a molecule of bacterial origin,” “cellular response to lipopolysaccharide,” “cellular response to molecule of bacterial origin,” and “regulation of DNA-binding transcription factor activity DNA” (Figures 2(a) and 2(b)). The results showed that the 10 network core genes primarily mapped to antiviral infection-related KEGG terms, such as “hepatitis B,” “human cytomegalovirus infection,” “hepatitis C,” “Kaposi sarcoma-associated herpesvirus infection,” “lipid and atherosclerosis,” “human T cell leukemia virus 1 infection,” and “Salmonella infection.”

### 3.3. Construction and Validation of the Lasso Regression Prediction Model

Then, the expression levels of 10 core genes in the drug-target network were differentially analyzed in normal and tumor cells. A heatmap (Figure 3(a)) and violin diagram (Figure 3(b)) of differential gene expression were drawn. Seven of the target core genes showed differential expression: *TP53* (*P* < 0.001), *MAPK1* (*P* < 0.001), *RELA* (*P* < 0.001), *CASP8* (*P* < 0.001), *MAPK3* (P < 0.001), *MYC* (*P* < 0.001), and *IL6* (*P* < 0.001), while the differences in *NFKBIA* (*P* = 0.859) and *NFKB1* (*P* = 0.312) expression were not statistically significant.

We conducted a coexpression correlation study and mapped the gene association (Figure 3(c)) to investigate whether there was a coexpression correlation among the seven differentially expressed drug-target network core genes. The coexpression of RELA and MAPK1 was the strongest, with a correlation coefficient of 0.58, showing a significant positive correlation.

Then, we performed univariate Cox prognostic regression analysis of the core network genes (Figure 3(d)). Among the 7 differentially expressed drug-targeting network core genes, 4 genes were associated with prognosis: *CASP8*, *MAPK1*, *MAPK3* and *RELA*. The results showed that these 4 drug-targeting network core genes were associated with prognosis. The remaining genes were not significantly associated with prognosis (*P* > 0.05), and the differences were not statistically significant. Next, the relationship between the expression levels of the four core genes of the drug target network and clinical survival was analyzed by the Lasso-Cox prognostic regression model, to construct a prognostic prediction model of multiple genes (Figures 3(e) and 3(f)). When *λ* = −0.389, the Lasso-Cox prognostic regression model had three prognostic model genes, namely, *CASP8*, *MAPK1*, and *MAPK3*, with regression coefficients of Coef(*CASP*8) = 0.04145626, Coef(*MAPK*1) = 0.05379257, and Coef(*MAPK*3) = 0.05630515. Therefore, the risk score formula for the sample was as follows: Risk score = 0.04145626∗*CASP*8 + 0.05379257∗*MAPK*1 + 0.05630515∗*MAPK*3.

The risk scores of all samples were calculated according to the risk score formula and stratified into high-risk and low-risk groups according to the median risk score, with a median risk value of 1.03967214. The risk score was calculated jointly with the survival status and survival time of the samples, and the high-risk and low-risk survival curves were obtained (Figure 3(g)). Likewise, patients in the high-risk group were more likely to encounter death earlier and had a poorer survival status than those in the low-risk group. The difference in prognosis between the two was statistically significant (*P* < 0.001). We plotted the ROC curve (Figure 3(h)) to verify the accuracy and reliability of the Lasso-Cox prognostic regression model's predictability. The ROC curve showed an AUC value of 0.718 (AUC value > 0.70), proving that Lasso-Cox's prognostic regression curve is reliable. We generated a risk curve (Figure 3(i)), risk, and survival scatter plot (Figure 3(j)). From the heatmap of model gene expression (Figure 3(k)), we found that patients in the high-risk group had a higher mortality probability and a higher gene expression level than those in the low-risk group. It is clear from the differential gene expression heatmap that the risk score can divide the model genes of the Lasso-Cox prognostic regression model into high- and low-risk groups. Thus, the risk score can clearly distinguish the gene expression, survival time, and survival status of high-risk and low-risk populations.

To validate the generality of the Lasso-Cox predictive regression model, we downloaded 442 transcriptomic data and clinical data of hepatocellular carcinoma samples from the Institute of Physical and Chemical Research of Japan (RIKEN, JP) in the ICGC database. Transcriptome data in the ICGC database and TCGA database were normalized. We combined gene expression and clinical data of tumor samples to plot survival curves related to risk values for the ICGC validation group, and the curves were divided into high- and low-risk groups (Figure 4(a)) (*P* < 0.05). The AUC of the ROC curve >0.6 indicated that the model was accurate (Figure 3(b)). The risk curve (Figure 4(c)), risk and survival scatter plots (Figure 4(d)), and heatmap of model gene expression in the high- and low-risk groups (Figure 4(e)) were significantly different. These results demonstrated the generalizability and accuracy of this Lasso-Cox predictive regression model. Both univariate prognostic analysis (Figure 4(f)) and multifactorial prognostic analysis (Figure 4(g)) were performed, and the risk values consistently correlated highly with sample survival status across a wide range of clinical data.

Both univariate prognostic analysis (Figure 4(f)) and multivariate prognostic analysis (Figure 4(g)) were performed, and the risk value consistently correlated highly with sample survival status across a wide range of clinical data.

A survival prognosis nomogram (Figure 4(h)) was plotted combining the risk score formula with survival to predict patient survival at 1-3 years in clinical practice.

We plotted the binding of glycyrrhizin to *CASP8* (Figure 4(i)) and the binding of matrine to *MAPK1* and *MAPK3* (Figures 4(j) and 4(k)), demonstrating the ability of matrine and glycyrrhizin to bind to target proteins to produce pharmacological effects.

### 3.4. Enrichment Analysis of the Model Gene GSEA Cellular Pathway

To investigate the positive correlation of genes of tumor-associated and immune-associated pathways in the Lasso-Cox prognostic regression model, we selected cellular pathways associated with tumorigenesis, development, and immune-related pathways for GSEA pathway-related enrichment analysis, and all pathways were screened by *P* < 0.05 significant difference (Figures 5(a)–5(c)). The *CASP8* and *MAPK1* genes had a strong correlation with 9 tumor-associated cellular pathways, but there was only one pathway difference between the two. *CASP8* was associated with the “ubiquitin-mediated proteolysis” pathway, while *MAPK1* was associated with the “transforming growth factor *β* signaling pathway.” The *MAPK3* gene was associated with four tumor-related cellular pathways: “cell cycle,” “DNA replication,” “pathways in tumors,” and “ubiquitin-mediated proteolysis.”

### 3.5. The Influence of Model Genes on Tumor Immunity

Next, we determined whether genes in the Lasso-Cox prognostic regression model influence the immune response. Immunoprediction data of HCC samples from the TCGA database were downloaded from the TIMER2.0 database. We plotted the histogram (Figure 5(d)), which showed the various immune cell contents in the samples, and the diagram of correlations between the levels of various immune cells (Figure 5(e)). The diagram of correlation showed that macrophage M0 cells had the smallest correlation -0.7 with T cells and CD8 cells. The correlation between memory CD4+ T cells and CD8+ T cells was highest at 0.49. Second, the correlation between the risk values and the content of various types of immune cells was studied, and scatter plots were drawn (Figures 5(f)–5(k)). As shown in the figure, six immune types of cells, including B cells, CD4 T cells, CD8 T cells, macrophages, dendritic cells, and neutrophils, were positively correlated with the risk score, and they were all statistically significantly different (*P* < 0.001). We then analyzed the correlation between risk values and various immune checkpoints (Figures 5(l)–5(q)). Risk values were strongly correlated with immune checkpoints (Figure 6(a)), and each immune checkpoint was also differentially expressed between normal and tumor samples (Figure 6(b)). Thus, it can be found that the risk score of the Lasso-Cox prognostic regression model is positively correlated with immune cells and is more strongly correlated with immune checkpoints. Scientists have recently begun investigating the function of nanoparticles in immunotherapy, for example, silica nanoparticles. Nanoparticle application in cancer is a field that is becoming increasingly promising [39].

### 3.6. Immunohistochemical Expression in the HPA Database

Immunohistochemical images downloaded from the HPA Human Protein Database (Figures 6(c), 6(d), 6(f), 6(g), 6(i), and 6(j)) showed that the immunofluorescent antibodies used in normal and tumor samples remained the same. IOD values were low-moderately expressed in normal tissues and moderately highly expressed in tumor tissues among the three model genes (Figures 6(e), 6(h), and 6(k)).

## 4. Discussion

Current treatments for cancer include surgery, radiotherapy, chemotherapy, targeted therapy, biotherapy, and complementary and alternative medicine (CAM) therapies such as traditional Chinese medicine (TCM) [40]. However, none of these approaches have achieved optimal efficacy without adverse events. Traditional single-target drug applications are insufficient to treat complex diseases such as cancer, cardiovascular disease, and Alzheimer's disease. TCM considers the body as a single complex system that is treated with Chinese herbal medicines (CHMs) and Chinese herbal formulas (CHFs) under the guidance of TCM theory. Each CHM is a mixture of multiple compounds. Many CHMs are biologically active, while individual substituents may not exhibit bioactivity, suggesting that multiple components of an herb have synergistic effects [41, 42]. In addition, in TCM, formulas are used more frequently. A formula usually consists of a larger number of herbs, which are systematically arranged in a hierarchical ranking. Therefore, synergistic combinations of CHMs alone or in combination with chemotherapeutic agents may be more suitable for the treatment of complex pathologies such as cancer. CHM compounds are bioactive, and studies on synergistic combinations of CHM compounds for the treatment of cancer have focused on combinations based on curcumin, quercetin, and resveratrol. For example, curcumin acts on the expression of tumor suppressor genes, apoptosis genes, oncogenes, and their respective proteins and signaling pathways [43]. Several CHM compounds have been combined with curcumin to enhance therapeutic efficacy. In vitro and in vivo studies have shown that the combination of curcumin and resveratrol enhances the apoptotic effects of head and neck cancer cells, including upregulation of PARP-1 cleavage and the Bax/Bcl-2 ratio and downregulation of ERK1 and ERK2 phosphorylation.

CHM combinations represent the core of CHFs. TCM physicians combine CHMs to enhance therapeutic effects and alleviate toxicity and side effects. Yanhusuo (Rhizoma corydalis) extract has been reported to weaken the invasive and metastatic ability of breast cancer cells. Furanodiene isolated from Ezhu (Rhizoma curcumae) has been shown to inhibit proliferation and apoptosis in lung cancer cells [44, 45]. Further studies on the synergistic effects of Ezhu and Yanhusuo showed that the 3 : 2 combination of Ezhu and Yanhusuo reduced the proliferation and invasive capacity of breast cancer cells more significantly than treatment with Ezhu and Yanhusuo alone and induced more cytochrome c release (initiation of apoptosis) [46]. The proper addition of CHM compounds, CHMs or CHFs enhances immunity and improves tolerance to chemotherapy, potentiates the cytotoxicity induced by chemotherapeutic drugs, and largely alleviates their side effects, ultimately improving patients' quality of life and prolonging their lifespan [47]. CHM compounds, CHMs or CHFs may significantly enhance the cytotoxic effects of chemotherapeutic agents. A prospective phase II study in patients with regressive or refractory multiple myeloma showed improved efficacy with the combination of melphalan with ascorbic acid and arsenic trioxide [48]. Alleviation of side effects is an important rationale for the use of CHMs in chemotherapy. The addition of Astragalus polysaccharide significantly alleviated the side effects of fatigue, nausea and vomiting, pain, and loss of appetite associated with the treatment of advanced NSCLC patients with vinorelbine and cisplatin, greatly improving the quality of life of patients [49].

Nevertheless, the concomitant use of CHM compounds, CHMs, or CHFs with or without chemotherapy might fail to achieve synergistic efficacy [50]. Moreover, not all combinations lack harmful effects [51]. In terms of combinations of CHM compounds, CHMs and CHFs, there is a large discrepancy between experimental data and clinical use. More efficient and reliable methods for researching and estimating the synergistic effects of CHM-related combinations should be optimized, such as the network-based approach and pharmacological networks [52]. In addition, studies of high quality, especially in the clinic, are needed. The role of the tumor-promoting inflammatory microenvironment and abnormal energy metabolism and its interference by herbs or herbal combinations should be highlighted.

In this study, we obtained 10 core drug-target network genes by analyzing the drug-target interaction network data of two extracted compounds from Chinese medicine: *TP53*, *CASP8*, *MAPK1*, *MAPK3*, *MYC*, *RELA*, *NFKB1*, *IL6*, and *NFKBIA*. There are many genes and key genes that affect tumor development, such as the NF-kappa B-cell pathway, MAPK/ERK signaling pathway, TNF (tumor necrosis factor) signaling pathway, IL-6 signaling pathway, TP53 signaling pathway and MYC signaling pathway, which are important cellular pathways in a variety of tumors.

Many studies have shown that matrine has anticancer properties. It treats or delays the onset and progression of tumors by inhibiting the cell division cycle, inducing apoptosis, and inhibiting the metastasis and proliferation of cancer cells. It can also reverse anticancer drug resistance and reduce anticancer drug side effects. These effects have enabled the widespread use of matrine for the treatment of various cancers and common types of cancer, such as lung, breast, stomach, esophagus, colon, liver, and pancreatic cancers. Matrine is often used as the main ingredient in injections to improve chemotherapy efficacy and reduce chemotherapy toxicity [53]. Matrine treatment destroys liver cancer cells through multiple ways. For example, matrine can promote apoptosis in HCC cells by triggering mitochondrial division and activating the Mst1-JNK signaling pathway, thereby triggering endogenous apoptosis [54]. Matrine activates the AMP protein kinase (AMPK) signaling pathway, inhibits p53 protein expression, and suppresses autophagy. Matrine inhibits the AMPK signaling pathway and converts autophagy into apoptosis [55]. When combined with sorafenib, matrine inhibits miR-21 while upregulating PTEN expression and inducing apoptosis in hepatocellular carcinoma cells [56]. Studies have shown that matrine and glycyrrhizin produce anticancer effects in vivo and in vitro, respectively [57, 58]. Both have the ability to protect the liver in cases of acute liver injury caused by various chemicals. Serological evidence [59, 60] suggested that matrine and glycyrrhizin could inhibit the precancerous stage of tumors and had a positive effect on tumor prevention.

Matrine reduces the activity of the ERK pathway by promoting the phosphorylation of MAPK1 and MAPK3 [61], thereby reducing the aggressiveness of HCC [62]. In this study, similar conclusions were also obtained through network pharmacology and various bioinformatics methods. Therefore, the anticancer effect of matrine may be closely related to the two genes. Matrine inhibits pancreatic cancer by inhibiting the NF-kappa B signaling pathway [61]. Matrine induces apoptosis of cancer cells by inhibiting the invasion and metastasis of pancreatic, prostate, and osteosarcoma tumors [62–64]. Matrine inhibits the expression of the MYC signaling pathway and has a growth inhibitory effect on human leukemia cells [65]. It inhibits the IL-6 cellular pathway and suppresses the expression of TNF, which has therapeutic effects on mouse colorectal cancer models. Matrine also inhibits the migration and proliferation of lung adenocarcinoma cells by upregulating TP53 expression levels. We consider that this effect may also occur in the treatment of hepatocellular carcinoma [66].

Studies have shown that glycyrrhizin has hepatoprotective, antiviral, anti-inflammatory, anti-immune, and antiulcer effects [67]. Research has also shown that glycyrrhizin has a protective effect against acute liver failure [60]. In addition, diammonium glycyrrhizinate subdues the severe symptoms of COVID-19, such as dyspnea, high fever (above 38 degrees Celsius), and confusion [68]. Emerging evidence has demonstrated that glycyrrhizin has potential antioxidative stress activity in vitro and in vivo (Figure 3). This study showed that glycyrrhizin could effectively inhibit the expression of CYP1A2 and CYP2E1 metabolic enzymes, thereby reducing the generation of the strong electronic active product trichloromethyl (·CC13) and inhibiting its occurrence from the beginning of the damage mechanism [69]. CYP1A2 and CYP2E1 are the main enzymes of the liver CYP enzyme system that metabolize exogenous substances [70], which are important targets involved in the regulation of CCL4-induced liver injury [71]. The increased expression of CYP1A2 and CYP2E1 can lead to a significant increase in the production of strong oxidative active metabolites by CCl4, thereby aggravating liver injury [72]. Mitochondria are the body's energy supply centers. Mitochondrial dysfunction can lead to mitochondrial oxidative stress, further amplifying its benefits, leading to the release of cytochrome C in mitochondria into the cytosol, further promoting the release of inflammatory factors, and then activating downstream molecular pathways, causing the occurrence of apoptosis. GLDH mainly exists in the mitochondrial matrix of hepatocytes. The significant increase in GLDH indicates that the mitochondria of liver cells are damaged, and a large amount of GLDH is released from mitochondria, leading to a significant increase in its content in blood [73]. In this study, matrine and glycyrrhizin were found to reduce the content of GLDH in the model group (*P* < 0.05), and the results indicated that both glycyrrhizin and matrine could restore mitochondrial energy metabolism and protect mitochondrial function. In addition, the results of serological tests also suggested that when the two drugs were combined, the effect was significantly better than that of single drug administration. In addition, glycyrrhizin, a commonly used HMGB1 inhibitor, significantly inhibited the expression of HMGB1 and thus c-MYC, thereby suppressing hepatocellular carcinoma [74].

Experimental studies in mice showed that the combination of matrine and glycyrrhizin significantly reduced the hepatotoxicity of acetaminophen in mice (*P* < 0.05). Compared with glycyrrhizin and matrine alone, the 48-hour mortality rate in mice was reduced by 20% and 26.7%, respectively, and the acetaminophen-induced increase in hepatic body mass ratio was significantly reduced. These results suggested that matrine and glycyrrhizin have protective effects on liver function. Moreover, the combination of matrine and glycyrrhizic acid increased the content of CD4+ and CD8+ immune cells in the peripheral blood of mice, indicating that their combination has the effect of regulating cellular immunity. The gut microbiota is important for the host's health and physiology. The gut microbiota and its metabolites may activate the immune response and cellular pathways that kill invading pathogens and initiate a cancer-fighting immune response [75–78]. The combination of matrine and glycyrrhizic acid can also enhance apoptosis and immune function and weaken the immunosuppression induced by cyclophosphamide (CTX). Combined application is better than glycyrrhizic alone. Studies have shown that the combination of matrine and glycyrrhizic acid can reduce the absorption of glycyrrhizic acid and accelerate its decomposition, thereby reducing the accumulation of glycyrrhizic acid in the body and reducing side effects such as sodium and water retention, hypertension, and hypokalemia caused by glycyrrhizic acid [79]. At the same time, studies have shown that the combined application has nonspecific anti-inflammatory effects [33].

Through analysis and mining, we obtained the drug-target interaction network of matrine and glycyrrhizin in the treatment of HCC. Although the combination of matrine and glycyrrhizin can enhance liver protection, anticancer, and nonspecific immunity and reduce immunosuppressive effects, side effects, and precancerous lesions, it is not clear whether the combination of the two components can increase the effectiveness and reduce the burden. The bioinformatics database provides bioinformation on the biomolecular action pathways and gene pathways of the two components of the core network of genes in vivo. In this study, we initially explored the molecular interaction mechanism of the two components in the treatment of HCC, which laid the foundation for further research on the mechanism of biomolecular action. In this study, we concluded that matrine and glycyrrhizin are effective in the combined treatment of HCC through gene functions, Gene Ontology such as “cellular response to biotic stimulus,” “cellular response to tumor necrosis factor,” “response to tumor necrosis factor,” “response to lipopolysaccharide,” “response to molecule of bacterial origin,” “cellular response to lipopolysaccharide,” “cellular response to molecule of bacterial origin,” “regulation of DNA-binding transcription factor activity,” “interleukin-1-mediated signaling pathway,” and “response to nicotine” as well as multiple KEGG cell pathways such as “hepatitis B,” “human cytomegalovirus infection,” “hepatitis C,” “Kaposi sarcoma-associated herpesvirus infection,” “lipid and atherosclerosis,” “human T cell leukemia virus 1 infection,” “Salmonella infection,” “IL-17 signaling pathway,” “Chagas disease,” “Toll-like receptor signaling pathway,” “C-type lectin receptor signaling pathway,” “TNF signaling pathway,” “apoptosis,” “influenza A,” “NOD-like receptor signaling pathway,” “pathogenic Escherichia coli infection,” and “Epstein–Barr virus infection.”

Matrine and glycyrrhizin have similar effects on many molecular pathways and gene functions, such as inhibition of the MAPK/ERK signaling pathway, IL-6 signaling pathway, tumor necrosis signaling pathway, nuclear factor-kappa B signaling pathway, TP53 signaling pathway, and MYC signaling pathway. In addition, glycyrrhizin, a common inhibitor of HMGB1, could reduce the level of CASP8 by decreasing the level of HMGB1, which has been experimentally shown to be an upstream gene of nuclear factor-kappa B, further reducing the activity of the nuclear factor-kappa B signaling pathway, thus demonstrating that glycyrrhizin could affect CASP8. Glycyrrhizin may exert effects and further inhibit cancer development through the CASP8-NF-kappa B pathway. It is noteworthy that glycyrrhizin affects CASP8, thus affecting the occurrence and development of tumors. Although there is no direct evidence yet, we look forward to follow-up pharmacological experiments [80]. However, through the molecular docking prediction diagrams of glycyrrhizin and CASP8, we also suspect that glycyrrhizin may have a direct drug-target interaction with CASP8, which may become a new finding in this study.

In addition, we performed Lasso-Cox regression analysis to construct a Lasso-Cox regression prognostic analysis model with risk scores for patients treated with two components or planned to use two components for HCC. We obtained the risk score and prognosis survival of the patients by this model. We could interpret the risk score and prognostic survival through the nomogram of this prognostic model to guide the clinical treatment strategy.

By analyzing the biological information of matrine and glycyrrhizin in the treatment of HCC, the risk value of matrine and glycyrrhizin was positively correlated with 6 immune cells. In addition, the differential expression boxplots were drawn by measuring the immunohistochemical gene expression levels between the tumor group and the normal group in the HPA database, which further verified the basic conclusion that the three risk genes were highly expressed in the tumor group (*P* < 0.05). Therefore, we believe that this prediction model is accurate. This study suggested that the same regimen of matrine combined with glycyrrhizin in the treatment of HCC may have better efficacy in patients with a higher risk value; that is, the level of immune cells in high-risk HCC patients may be higher than that in low-risk patients, and the expression of immune checkpoints is more obvious. Therefore, the risk values derived from this model may be useful to guide clinical immunotherapy. In the HCC tumor microenvironment, the immunosuppression of high-risk tumors may be stronger than that of low-risk tumors. Matrine and glycyrrhizin therapy may be beneficial for tumor immunotherapy in patients with HCC in clinical application.

## 5. Conclusions

Overall, this study analyzed the interactions and molecular mechanisms of the two drugs on HCC, confirming that the two drug components of matrine and glycyrrhizin do have synergistic effects. For example, both components have similar effects and can affect the NF-kappa B-cell, MAPK/ERK signaling, TNF signaling, IL-6 signaling, TP53 signaling, and MYC signaling pathways. Therefore, it is reasonable to believe that matrine and glycyrrhizin can synergize at the molecular pathway level.

Compared with previous studies, we used modern network pharmacology theory to analyze the molecular biological mechanism of matrine and glycyrrhizin in HCC, innovatively developed a Lasso-Cox prognostic regression model, and analyzed the immune effects of both drugs. These studies may be helpful to guide clinical practice. In future studies, we hope to verify the conclusions drawn from this study through pharmacological experiments and related molecular biology experiments to make the conclusions more accurate and reliable. There are still some areas to be improved upon in this study, which are expected to be supplemented in future studies.

## Figures and Tables

**Figure 1:** (a) Five disease gene databases combined with Venn diagrams. (b) Venn diagram of the intersection of drug targets and hepatocellular carcinoma genes. (c) Drug target interaction network. (d) Protein–protein interaction. (e, f) Screening network core genes.

**Figure 2:** (a, b) GO bubble and circle graphs of network core genes. (c, d) Bubble and circles of KEGG pathway of network core genes.

**Figure 3:** (a) Heatmap of network core gene expression in the TCGA database. (b) Violin diagram of differential expression of network core genes. (c) Correlation diagram of network core gene expression level. (d) Unigenic Cox prognostic regression analysis of network core genes. (e, f) Lasso prognostic regression model. (g) Survival curves in the TCGA database. (h) ROC curve to verify the accuracy of risk. (i) Risk curve. (j) Risk and survival scatter plot. (k) Heatmap of model gene expression in the high- and low-risk groups.

**Figure 4:** (a) Survival curve in the ICGC database. (b) ROC curve to verify the accuracy of risk. (c) Risk curve. (d) Risk and survival scatter plot. (e) Heatmap of model gene expression in the high- and low-risk groups. (f) Univariate prognostic regression test. (g) Multivariate prognostic regression test. (h) Used to predict survival in patients with the nomogram. (i, j, k) Panel (i) shows the predicted binding pattern of glycyrrhizin and CASP8 protein, and panels (j) and (k) show the predicted binding pattern of matrine to MAPK1 and MAPK3 proteins.

**Figure 5:** (a, b, c) GSEA enrichment analysis of CAPS8, MAPK1, and MAPK3, respectively. (d) Histogram of various immune cell contents in the TCGA database. (e) Diagram of correlations between the levels of various immune cells. (f, g, h, i, j, k) A linear regression diagram of various immune cell levels and risks. (l, m, n, o, p, q) Graph of linear regression between expression levels of various immune checkpoints and risk.

**Figure 6:** (a) Graph of the correlation between expression levels of various immune checkpoints. (b) Box plot of expression differences of various immune checkpoints between normal and tumor samples. (c, d) Immunohistochemical section images of CASP8 differentially expressed in normal and hepatocellular carcinoma tissues from the HPA database. (f, g) Immunohistochemical section images of MAPK1 differentially expressed in normal and hepatocellular carcinoma tissues from the HPA database. (i, j) Immunohistochemical section images of MAPK3 differentially expressed in normal and hepatocellular carcinoma tissues from the HPA database. (e, h, k) The boxplots of IOD differences of CASP8, MAPK1, and MAPK3 in normal tissues and tumor tissues, respectively.

## Data Availability

All the data can be obtained from the corresponding author upon request.
